# Long noncoding RNA ZNF667‐AS1 reduces tumor invasion and metastasis in cervical cancer by counteracting microRNA‐93‐3p‐dependent PEG3 downregulation

This article has been retracted.

**DOI:** 10.1002/1878-0261.12565

**Published:** 2019-10-17

**Authors:** Yong‐Jie Li, Zhe Yang, Yi‐Ying Wang, Yue Wang

**Affiliations:** ^1^ Department of Obstetrics and Gynecology Henan Provincial People's Hospital People's Hospital of Zhengzhou University Henan University People's Hospital China

**Keywords:** cervical cancer, invasion, metastasis, microRNA‐93‐3p, paternally expressed gene 3, zinc finger protein 667‐antisense RNA 1

## Abstract

Zinc finger protein 667‐antisense RNA 1 (ZNF667‐AS1), located on human chromosome 19q13.43, is a member of the C2H2 zinc finger protein family. Herein, we aimed to analyze the interactions between ZNF667‐AS1, microRNA‐93‐3p (miR‐93‐3p), and paternally expressed gene 3 (PEG3) and to explore their roles in the tumorigenesis of cervical cancer (CC). Differentially expressed long noncoding RNAs and miRNAs related to CC were determined using gene expression datasets sourced from the Gene Expression Omnibus database. Subsequently, the regulatory relationships between ZNF667‐AS1 and miR‐93‐3p and between miR‐93‐3p and PEG3 were identified using the dual‐luciferase reporter gene assay. In addition, the expression of miR‐93‐3p and ZNF667‐AS1 was up‐ or downregulated in CC cells (HeLa), in order to assess their effects on cell cycle distribution and cell invasion *in vitro*, and tumor growth and metastasis *in vivo*. MiR‐93‐3p was found to be highly expressed, while ZNF667‐AS1 and PEG3 were poorly expressed in CC. ZNF667‐AS1 could competitively bind to miR‐93‐3p, which targeted PEG3. In addition, miR‐93‐3p downregulation and ZNF667‐AS1 overexpression led to increased expression of PEG3, tissue inhibitor of metalloproteinases, and p16 and decreased expression of cyclin D1, matrix metalloproteinase‐2 and ‐9. MiR‐93‐3p inhibition and ZNF667‐AS1 elevation also inhibited cell cycle entry and cell invasion *in vitro*, but repressed tumor growth and metastasis *in vivo*. These key findings demonstrated that upregulation of ZNF667‐AS1 could suppress the progression of CC *via* the modulation of miR‐93‐3p‐dependent PEG3, suggesting a potential therapeutic target for the treatment of CC.

**Abbreviations**
CC: cervical cancer
GEO: Gene Expression Omnibus
HPV: human papillomavirus
lncRNAs: long noncoding RNAs
miR‐93‐3p: microRNA‐93‐3p
MMP‐2: matrix metalloproteinase‐2
MMP‐9: matrix metalloproteinase‐9
mRNAs: messenger RNAs
Mut: mutant type
NC: negative control
PEG3: paternally expressed gene 3
PI: propidium iodide
RT/qPCR: reverse transcription/quantitative PCR
TIMP‐2: tissue inhibitor of metalloproteinases‐2
Wt: wild type
ZNF667‐AS1: zinc finger protein 667‐antisense RNA 1

## 1 Introduction

Cervical cancer (CC) has been ranked as the second leading cause of cancer‐induced mortality in women worldwide; the incidence of CC is predominantly in developing countries where access to high‐quality healthcare systems that facilitate timely screening that facilitates early diagnosis of CC may be limited (Berman and Schiller, 2017). Another serious concern is that the overall rate of 5‐year survival for CC is relatively low (Li *et al.*, 2017). Epidemiologically, viral infections [e.g., human papillomavirus (HPV) infection] and early age of first sexual intercourse or first pregnancy have been associated with increased incidence and mortality of CC (Chetty, 2017; Louie *et al.*, 2009). Hysterectomy is one of the most widely adopted therapeutic approaches for managing patients with early‐stage CC, along with concurrent radiation and chemotherapy (Johansen *et al.*, 2016; Ross Green *et al.*, 2017). However, majority of CC treatment protocols confer to a poor prognosis in patients, particularly in those who underwent hysterectomy (Shim *et al.*, 2018). The molecular underpinnings of CC are not yet well elucidated. A deeper understanding of molecular mechanisms underlying CC occurrence and progression can aid the discovery of novel molecular therapeutic targets for its treatment.

Long noncoding RNAs (lncRNAs) are a group of non‐protein‐coding transcripts with lengths of 200 or more nucleotides, which function as important mediators in tumor development and progression (Yang *et al.*, 2014). LncRNAs are involved in the modulation of genes at transcriptional, post‐transcriptional, and chromosomal levels during various vital biological functions (Cao *et al.*, 2017). LncRNAs can modulate gene expression by binding to chromatin regulators and interfering with the functions of RNAs, thereby exercising their effects on cellular responses (Liao *et al.*, 2016). Zinc finger protein 667 (ZNF667) is an lncRNA capable of regulating numerous cellular processes, such as cell proliferation, migration, and invasion (Cheng *et al.*, 2017). ZNF667‐antisense RNA 1 (ZNF667‐AS1) is documented as a biomarker and a potential therapeutic target for CC (Zhao *et al.*, 2017). In general, the interaction of zinc finger proteins with microRNAs during cancer progression has been investigated in several recent studies (Hu *et al.*, 2018; Uchida *et al.*, 2014). As a class of small noncoding RNAs, microRNAs (miRNAs) play significant roles in post‐transcriptional gene regulation by targeting the 3′UTR of target messenger RNAs (mRNAs) and decreasing the stability and/or translation of these mRNAs (Bei *et al.*, 2016). MiRNA dysregulation and its effects have been observed in a variety of human diseases, and various miRNAs can function as potential candidates for CC treatment and prognosis (Liang *et al.*, 2017; Wang *et al.*, 2017; Zhou *et al.*, 2017). In particular, miR‐93 is reported to be involved in CC metastasis and invasion (Wang *et al.*, 2013). miRNAs‐93‐3p (MiR‐93‐3p) is shown to regulate the expression of RUNX2 gene by binding to its respective 3′UTR (Peng *et al.*, 2018). Paternally expressed gene 3 (PEG3) functions as an imprinted gene to encode a zinc finger DNA‐binding protein (He *et al.*, 2016). PEG3 is known to be epigenetically affected in several cancers, including CC, where it may act as a potential tumor suppressor (Nye *et al.*, 2013). However, the potential interactions between ZNF667‐AS1/miR‐93‐3p/PEG3 during the progression of CC remain largely unknown. To address this gap, the present study aimed to explore the regulatory network of ZNF667‐AS1/miR‐93‐3p/PEG3 in the invasion and metastasis of CC, with a view to generate insights into molecular mechanisms underlying CC and provide basis for new therapeutic targets.

## 2 Materials and methods

### 2.1 Ethics statement

The protocols of the present study were approved by the Ethics Committee of Henan Provincial People's Hospital, People's Hospital of Zhengzhou University, Henan University People's Hospital, and in accordance with the ethical standards formulated in the Declaration of Helsinki. All participating patients signed a written informed consent form prior to inclusion in the study. All animal experiments were performed in accordance with the guidelines issued in the Guide for the Care and Use of Laboratory Animal by the National Institutes of Health and with the approval of the Ethics Committee of Henan Provincial People's Hospital, People's Hospital of Zhengzhou University, Henan University People's Hospital.

### 2.2 Microarray‐based gene expression profiling

The Gene Expression Omnibus (GEO) database (http://www.ncbi.nlm.nih.gov/geo) was used to retrieve gene expression datasets and annotation, pre‐existing data related to CC. The sequencing results of Affymetrix™ U133A Plus 2.0 platform (Thermo Fisher Scientific, Waltham, MA, USA) were selected from the GSE26787 expression dataset. In addition, the remaining three gene expression datasets (GSE63514, GSE63678, and GSE9750) including the CC and normal samples were obtained from the GEO database. The Bioconductor ‘Affy’ package in the r software was employed for background correction and normalization of the gene expression datasets (Fujita *et al.*, 2006). Subsequently, linear models with empirical Bayes method from the Limma package were applied in conjunction with traditional *t*‐tests, in order to filter nonspecific noise from the expression data and screen differentially expressed mRNAs and lncRNAs (Smyth, 2004).

### 2.3 Study subjects

Cervical cancer tissues and adjacent normal tissues were collected from 64 patients pathologically diagnosed with CC and undergoing radical resection in the Henan Provincial People's Hospital, People's Hospital of Zhengzhou University, Henan University People's Hospital, from August 2014 to May 2017. The enrolled patients were aged between 29 and 67 years. They included 43 cases of squamous cell carcinomas and 21 cases of adenocarcinoma. The clinical stage of CC was assigned according to the classification criteria recommended by the International Federation of Gynecology and Obstetrics (2016). Among the enrolled patients, there were eight cases of stage I, 14 cases of stage II, 23 cases of stage III, and 19 cases of stage IV CC.

### 2.4 Reverse transcription/quantitative PCR (RT/qPCR)

Reverse transcription/quantitative PCR (RT/qPCR) analysis was applied to the specimens of CC and adjacent normal tissues. Total RNA from tissues and cells was extracted using a Trizol Kit (15596026; Invitrogen Inc., Carlsbad, CA, USA). miRNA was extracted using a mirVana miRNA isolation kit (AM1552; Ambion Inc., Carlsbad, CA, USA). A DU‐640 spectrophotometer (Beckman Coulter, Inc., Brea, CA, USA) was employed to determine the concentration and purity of the extracted RNA (a ratio of A_260_/A_280_ between 1.8 and 2.0 was considered as high purity). The RNA was then reverse‐transcribed into cDNA in accordance with the instructions of a PrimeScript RT reagent Kit (RR047A; Takara Bio, Tokyo, Japan). RT/qPCR was performed in an ABI7500 instrument (Applied Biosystems, Inc., Carlsbad, CA, USA) using a SYBR Premix EX Taq Kit (Takara Biotechnology Ltd., Dalian, China). Primer sequences (Table 1) were synthesized by Shanghai Genechem Co., Ltd. (Shanghai, China). U6 was set as the internal reference for miR‐93‐3p and glyceraldehyde‐3‐phosphate dehydrogenase (GAPDH) was set as the internal reference gene for other transcripts. The 2^−ΔΔCt^ method (ΔΔCT = ΔCt_experimental group_ − ΔCt_control group_, and ΔCt = Ct_target gene_ − Ct_internal reference_) was used to calculate the relative mRNA expression of each target gene. Each biological sample was run in triplicate and experiments were independently repeated thrice.

**Table 1:** Primer sequences of ZNF667‐AS1, miR‐93‐3p, PEG3, MMP‐2, MMP‐9, TIMP‐2, P16, and cyclin D1 for RT/qPCR.

Gene	Sequence	Amplification product length (bp)
ZNF667‐AS1 (NR_036521.1)	F: 5′‐GGGAGTGTCCGCCATAAAGT‐3′	195
	R: 5′‐AGATCGTAGCAGGGTCCAGT‐3′	
miR‐93‐3p (MIMAT0004509)	F: 5′‐TCGGCAGGACTGCTGAGCTAGC‐3′	52
	R: 5′‐CTCAACTGGTGTCGTGGA‐3′	
PEG3 (NM_001146184.1)	F: 5′‐CCTACCCAAGCACCAGTCG‐3′	137
	R: 5′‐GGAACTGCGTGACACATCCT‐3′	
MMP‐2 (NM_004530.5)	F: 5′‐AGATCTTCTTCTTCAAGGACCGGTT‐3′	225
	R: 5′‐GCGGAGATTGGGAACCAGCTGTA‐3′	
MMP‐9 (NM_004994.2)	F: 5′‐GCGGAGATTGGGAACCAGCTGTA‐3′	209
	R: 5′‐GACGCGCCTGTGTACACCCACA‐3′	
TIMP‐2 (S48568.1)	F: 5′‐AAACGACATTTATGGCAACCCTATC‐3′	430
	R: 5′‐ACAGGAGCCGTCACTTCTCTTGATG‐3′	
P16 (NM_058195.3)	F: 5′‐GGGTTTTCGTGGTTCACATCC‐3′	105
	R: 5′‐CTAGACGCTGGCTCCTCAGTA‐3′	
Cyclin D1 (BC023620.2)	F: 5′‐GCTGCGAAGTGGAAACCATC‐3′	135
	R: 5′‐CCTCCTTCTGCACACATTTGAA‐3′	
U6 (NR_004394.1)	F: 5′‐GCTTCGGCAGCACATATACTAAAAT‐3′	89
	R: 5′‐CGCTTCACGAATTTGCGTGTCAT‐3′	
GAPDH (NM_002046.6)	F: 5′‐GGTGAAGGTCGGAGTCAACGG‐3′	69
	R: 5′‐CCAGAGTTAAAAGCAGCCCTGG‐3′	

### 2.5 Cell transfection

After regular recovery, HeLa and C‐33A cells were cultured in a 5% CO_2_ incubator (BB15; Thermo Fisher Scientific Inc., Waltham, MA, USA) at 37 °C and saturated humidity in Dulbecco’s modified Eagle’s medium (DMEM, 12800017; Gibco BRL, Grand Island, NY, USA) supplemented with 10% FBS. Upon 90% cell confluence, a subculture was performed. Cells from the third passage in the logarithmic growth phase were treated with 0.25% trypsin and DMEM supplemented with 10% FBS to obtain a single‐cell suspension. The cell suspension was assigned into 10 groups of transfection: the control group (no transfection), the vector group (transfected with positive control plasmid), the ctrl siRNA group [transfected with negative control (NC) plasmid], the ZNF667‐AS1 vector group (transfected with pcDNA‐ZNF667‐AS1), the si‐ZNF667‐AS1 group (transfected with anti‐ZNF667‐AS1 siRNA), the miR‐93‐3p mimic group (transfected with miR‐93‐3p mimic), the NC‐mimic group (transfected with NC plasmid for miR‐93‐3p mimic), the miR‐93‐3p inhibitor group (transfected with miR‐93‐3p inhibitor), the NC inhibitor group (transfected with NC plasmid for miR‐93‐3p inhibitor), and the si‐ZNF667‐AS1 + miR‐93‐3p inhibitor group (cotransfected with anti‐ZNF667‐AS1 siRNA and miR‐93‐3p inhibitor).

### 2.6 Fluorescence *in situ* hybridization (FISH)

Fluorescence *in situ* hybridization (FISH) was performed in order to identify the subcellular localization of ZNF667‐AS1 in CC cells. HeLa and C‐33A cell slides were treated with Proteinase K solution (200 μL·mL^−1^) at 37 °C for 5 min and then immersed in HCL (0.1 mol·L^−1^) for 10 min at room temperature. Subsequently, the slides were dehydrated with an alcohol gradient of 70%, 85%, and 100% and heated at 56 °C for 5 min. The cell slides were successively treated with a 10 μL mixture of hybridization buffer, ZNF667‐AS1 probe (synthesized by Sangon Biotech Co., Ltd., Shanghai, China), and deionized water in conditions devoid of light. These were then denaturized at 83 °C for 10 min using an *in situ* hybridization apparatus. After incubating the slides at 37 °C overnight, the cover slip was removed and the cells were stained with 15 μL of 4′,6‐diamidino‐2‐phenylindole (DAPI) for 10–20 min in the dark. Finally, the samples were observed under a fluorescence microscope.

### 2.7 Transwell assay

After 48 h of transfection, the cells were fasted in serum‐free medium for 24 h. Following trypsinization, the cells were suspended in serum‐free Opti‐MEMI (Invitrogen) supplemented with bovine serum albumin (10 g·L^−1^) and adjusted to a density of 3 × 10^4^ cells·mL^−1^. Transwell assay was conducted in a 24‐well Transwell plate (8 μm pore size; Corning Inc., Corning, NY, USA) by seeding 100 μL of cell suspension into each well, with triplicate repetition in each group. Next, 600 μL of DMEM containing 10% FBS was added to each basolateral chamber and the Transwell plate was incubated at 37 °C under 5% CO_2_. Matrigel (50 μL) was then fully coated on the chambers. After 24 h of cell culture, the Transwell chamber was removed and the bottom of the basolateral chamber was repeatedly washed with the culture medium in the basolateral chamber. Cells on the apical layer of the polycarbonate membrane were wiped away with a cotton swab, and fluorescent cells adhering to the basolateral layer of the chamber were immediately observed under an inverted fluorescence microscope. Five visual fields were randomly selected for cell counting, and the mean number of cells that had crossed through the Matrigel was determined. The results were considered indicative of the cell invasion ability. Each experiment was repeated three times.

### 2.8 Flow cytometry

Propidium iodide (PI) single staining was adopted for analyzing the cell cycle distribution. After 48 h of transfection, the cells were treated with 0.25% trypsin and prepared into a single‐cell suspension. The cells were then treated with 20 μL RNase for 30 min at 37 °C and stained with PI (400 μL) on ice for 15 min, avoiding exposure to light. The cell cycle distribution was analyzed by flow cytometry at an excitation wavelength of 488 nm. Mean values determined from three independent experiments were recorded.

### 2.9 Dual‐luciferase reporter gene assay

A web‐based bioinformatic prediction resource (https://cm.jefferson.edu/rna22/Interactive/) was used to predict the binding sites of miR‐93‐3p on ZNF667‐AS1 and PEG3 each. PCR was then applied for amplification of the ZNF667‐AS1 sequence in its 3′UTR region. The target fragment was cloned into the downstream of pmirGLO (3577193; Promega Corp., Madison, WI, USA) using the Xho I and Not I restriction sites. The obtained recombinant plasmid [pZNF667‐AS1‐wild type (Wt), CGAGGAGGGGCGGACAGCGGA] was then purified using bacterial culture and stored for subsequent experiments. Site‐specific mutagenesis was performed on the miR‐93‐3p binding site of ZNF667‐AS1 to construct a pZNF667‐AS1‐mutant type (Mut) plasmid (ACTGCTGAGCTAGCACTTCCCG). Luciferase reporter gene assay was employed to validate whether PEG3 was a direct target of miR‐93‐3p. PEG3 was inserted into a pMIR reporter between two restriction sites (Spe I and Hind III, namely pPEG3‐Wt (TGGGGAGTGCTTGCTCATAGC). A complementary sequence mutation site of the seed sequence was designed based on Wt PEG3. The target fragment was subsequently inserted into the pMIR reporter plasmid using T4 DNA ligase, namely pPEG3‐Mut (ACTGCTGAGCTAGCACTTCCCG). The correct luciferase reporter plasmids of Wt and Mut miR‐93‐3p were cotransfected into HEK‐293T cells (CRL‐1415; Shanghai Xin Yu Biotech Co., Ltd., Shanghai, China). Following 24 h of transfection, the cells were lysed and centrifuged at 16000 *g* for 1 min to collect the cell supernatant. The Dual‐Luciferase^®^ Reporter Assay System (E1910; Promega Corp.) was utilized to measure luciferase activity in the transfected cells by adding a combination of 100 μL of firefly luciferase working solution and 100 μL of Renilla luciferase working solution into each sample. The relative luciferase activity was expressed as the ratio of firefly luciferase activity to Renilla luciferase activity. Each experiment was repeated three times.

### 2.10 RNA pull‐down assay

Sequences of Bio‐probe‐NC (AACGUGGCUACCGUAGUAUUGC), Bio‐miR‐93‐3p‐Wt (CGGGAAGUGCUAGCUCAGCAGU), ZNF667‐AS1‐Wt (CGAGGAGGGGCGGACAGCGGA), ZNF667‐AS1‐Mut (AGTCAATGCAGAGTTAGTCGT), Bio‐miR‐93‐3p‐Mut (UGGGGAGUGCUUUGCUCAUAGC), PEG3‐Wt (TGGGGAGTGCTTTGCTCATAGC), and PEG3‐Mut (GCCATAGACCACGGATGTTAAG) were synthesized *in vitro* by Shanghai Sangon Biotechnology Co., Ltd., and then labeled using Biotin RNA Labeling Mix. The DNAs were treated with RNase‐free DNase I and purified using an RNeasy® Mini Kit (Qiagen, Hilden, Germany). The labeled RNA (1 μg) was heated in an RNA structure buffer (10 mmol·L^−1^ Tris pH 7, 0.1 mol·L^−1^ KCl, 10 mmol·L^−1^ MgCl_2_) to 95 °C for 2 min, incubated on ice for 3 min, and then incubated at room temperature for 30 min to allow the formation of a secondary structure. HeLa and C‐33A cells (3 μg) were lysed with a cell lysis buffer (Sigma‐Aldrich, St. Louis, MO, USA) at 4 °C for 1 h and centrifuged at 12 000 r.p.m. for 10 min. The supernatant was then collected, transferred to an RNase‐free centrifuge tube, washed twice with a combination of a low salt and a high‐salt buffer each (10 min each), and incubated with 500 μL of streptavidin–agarose beads for 1 h. After washing with a RIP buffer 5 times, RT/qPCR was performed in order to analyze the relationship between ZNF667‐AS1 and miR‐93‐3p.

### 2.11 Western blot analysis

Total protein was extracted from tissues and cells using a RIPA lysis buffer (R0010, Solarbio Science and Technology Corporation, Beijing, China) containing phenylmethanesulfonyl fluoride. The total protein concentration was evaluated using a bicinchoninic acid protein kit (23225; Pierce, Rockford, IL, USA). The obtained proteins were isolated using 10% sodium dodecyl sulfate/polyacrylamide gel electrophoresis (P0012A; Beyotime Institute of Biotechnology, Shanghai, China) and transferred onto polyvinylidene fluoride membranes. After being blocked with Tris‐buffered saline–Tween 20 containing 5% skimmed milk for 2 h, the proteins were incubated at 4 °C overnight with the following primary antibodies: rabbit anti‐PEG3 (1:1000, ab196738), anti‐matrix metallopeptidase (MMP)‐2 (1 μg·mL^−1^, ab37150), anti‐MMP‐9 (1 μg·mL^−1^, ab73734), antitissue inhibitor of metalloproteinases‐2 (TIMP‐2; 1:1000, ab1828), anti‐p16 (1:1000, ab151303), anti‐cyclin D1 (1:1000, ab16663), and anti‐GAPDH (1:2500, ab9485; Abcam Inc., Cambridge, MA, USA). Next, the proteins were incubated with horseradish peroxidase‐conjugated goat anti‐rabbit immunoglobulin G secondary antibodies (1:2000, ab6721, Abcam Inc.) at room temperature for 2 h. The membranes were then visualized using an enhanced chemiluminescence reagent (WBKLS0100; Millipore, Billerica, MA, USA). The gray value ratio of target protein to the internal reference GAPDH was determined and considered as the relative protein expression.

### 2.12 Tumor xenograft implantation in nude mice

BALB/c female nude mice (age: 44 weeks) were randomly grouped into control, ZNF667‐AS1 vector, si‐ZNF667‐AS1, and si‐ZNF667‐AS1 + miR‐93‐3p inhibitor groups, with 8 mice in each group. After transfection, the cells were subcutaneously implanted into the back of each nude mouse (5 × 10^6^ cells per mouse). The length and width of xenograft tumors were recorded every 3 days and used to calculate the tumor volume according to the formula: volume = (length × width^2^)/2. A growth curve was drawn using the volume of the transplanted tumors, and after 15 days, the nude mice were sacrificed. After dissection, the location and number of metastatic lymph nodes in the neck, axillary, abdominal aorta, groin, and areas surrounding the viscera were observed and recorded.

### 2.13 Immunohistochemistry assay

An immunohistochemistry assay was employed to measure the expression of metastasis‐associated protein 1 (MTA1) in the xenograft tissues. The xenograft tumor tissues were fixed in 4% neutral‐buffered formaldehyde (DF0113; Solarbio Science and Technology Corporation), embedded in paraffin, and dissected into multiple sections (4 μm in thickness). The sections were then baked at 60 °C for 1 h, deparaffinized in xylene (YB‐5485; Shanghai Yubo Biological Technology Co., Ltd., Shanghai, China), and dehydrated using the gradient alcohol. The sections were next incubated with 3% H_2_O_2_ at 37 °C for 30 min, blocked with 10% goat serum for 15 min, and incubated with rabbit anti‐MTA‐1 (1:1000, ab71153; Abcam Inc.) primary antibodies overnight at 4 °C. The sections were then incubated with the biotin‐conjugated goat anti‐rabbit secondary antibodies (1:1000, ab6721; Abcam Inc.) at 37 °C for 40 min and stained with diaminobenzidine (DA1010; Solarbio Science and Technology Corporation) for 10 min. Subsequently, the sections were counter‐stained with hematoxylin (H8070, Solarbio Science and Technology Corporation) for 1 min, dehydrated using gradient alcohol, dried, cleared in xylene, and mounted in neutral gum. Brownish‐yellow granules in the cytoplasm or on the cell membrane were considered indicative of positive MTA1 signals. During analysis, 10 visual fields were randomly selected on each section and the staining intensity was scored using the Breasalier method and the following criteria: Cells without coloration were considered as negative (0 point); yellowish coloration was considered as weakly positive (1 point); brownish‐yellow coloration was considered as moderately positive (2 points); and brown coloration was considered as strongly positive (3 points). Upon counting the number of fields for each intensity, the mean intensity score (IS) was calculated based on the formula: IS = ∑ (0 × F0 + 1 × F1 + 2 × F2 + 3 × F3), where F denoted the number of cells in each field (at 10 × magnification) (Eilstein *et al.*, 2002).

### 2.14 *In situ* hybridization

Paraffin‐embedded sections were deparaffinized in water and detached with a 0.8% mixture of pepsin and hydrochloric acid at 37 °C for 10 min. The sections were washed with Tris‐buffered saline (TBS), dehydrated with gradient ethanol, and dried at room temperature. Subsequently, the sections were added with the probe and covered by a slide, followed by 10‐min denaturation at 98 °C and 1‐h hybridization at 37 °C. Next, the sections were washed with TBS, incubated with alkaline phosphatase‐labeled digoxin antibody at room temperature for 30 min, and visualized with 5‐bromo‐4‐chloro‐3‐indolyl phosphate/nitroblue tetrazolium in the dark. The visualization was controlled by observation under a microscope. Lastly, the sections were stained with 0.3% nuclear fast red, dehydrated, permeabilized, and mounted (Nose *et al.*, 2012; Shi *et al.*, 2009).

### 2.15 Statistics

Statistical analysis was performed using the spss 21.0 software (IBM Corp., Armonk, NY, USA). Measurement data were expressed as mean ± standard deviations. All experiments were conducted in triplicate. The data between CC and adjacent normal tissues were compared using paired *t*‐test. Comparisons between multiple groups were performed by one‐way analysis of variance (ANOVA), followed by Tukey *post hoc* test. Comparison of tumor volume in different mice was analyzed by repeated measurement ANOVA. A Pearson’s correlation test was employed for correlation analysis. A *P* value of < 0.05 was considered indicative of a significant statistical difference.

## 3 Results

### 3.1 ZNF667‐AS1 and PEG3 are poorly expressed while miR‐93‐3p is highly expressed in CC tissues

In order to identify lncRNAs that are differentially expressed in CC, we performed a comprehensive lncRNA profiling analysis using the GEO datasets (GSE27678, GSE63514, GSE63678, and GSE9750). Through analysis of microarray data (GSE27678 and GSE63514), expression of ZNF667‐AS1 and PEG3 was found to be downregulated in CC (Fig. 1A,B). PEG3 was noted to be downregulated in CC by the analysis of microarray datasets GSE63678 and GSE9750 (Fig. 1C,D). Bioinformatic analysis predicted a binding site of miR‐93‐3p in ZNF667‐AS1 (Fig. 1E) as well as in PEG3 (Fig. 1F). The expression of ZNF667‐AS1, miR‐93‐3p, and PEG3 was subsequently determined in resected CC versus adjacent normal tissues, using RT/qPCR. The expression of ZNF667‐AS1 and PEG3 was markedly reduced, while the expression of miR‐93‐3p was significantly increased in CC tissues as compared with adjacent normal tissues (Fig. 1G). ZNF667‐AS1 expression was negatively correlated with that of miR‐93‐3p but positively correlated with that of PEG3, while miR‐93‐3p expression was negatively correlated with PEG3 (Fig. 1H). These results signified that ZNF667‐AS1 and PEG3 were poorly expressed, while miR‐93‐3p was highly expressed in CC affected tissues.

**Figure 1:** MiR‐93‐3p expression was significantly increased, while the expression of ZNF667‐AS1 and PEG3 was decreased in CC tissues. (A) Heatmaps with hierarchical clustering analysis on the microarray dataset GSE27678 showed differentially expressed lncRNAs and genes. (B) Heatmaps with hierarchical clustering analysis on the microarray dataset GSE63514 showed differentially expressed lncRNAs and genes. (C) Heatmaps with hierarchical clustering analysis on the microarray dataset GSE63678 showed differentially expressed genes. (D) Heatmaps with hierarchical clustering analysis on the microarray dataset GSE9750 showed differentially expressed genes. (E) Website ‘RNA22’ was used to predict the binding site of miR‐93‐3p in ZNF667‐AS1. (F) Website ‘RNA22’ was used to predict the binding site of miR‐93‐3p in PEG3. (G) RT/qPCR revealed that ZNF667‐AS1 and PEG3 were poorly expressed while miR‐93‐3p was highly expressed in CC tissues. The data were expressed as mean ± standard deviation, conformed to normal distribution, and compared by paired *t*‐test. (H) Correlation between expression levels of ZNF667‐AS1, miR‐93‐3p, and PEG3 in CC tissues using Pearson’s correlation test. *n* = 64. *P < 0.05, CC tissues vs. the adjacent normal tissues.

### 3.2 PcDNA‐ZNF667‐AS1, si‐ZNF667‐AS1, miR‐93‐3p mimic, and miR‐93‐3p inhibitor were successfully transfected into HeLa and C‐33A cells

MiR‐93‐3p mimic and inhibitor were transfected into HeLa or C‐33A cells. In contrast to the HeLa cells without transfection, the cells transfected with miR‐93‐3p mimic presented with significantly increased miR‐93‐3p expression while the cells transfected with miR‐93‐3p inhibitor showed significantly decreased miR‐93‐3p expression (both *P* < 0.05, Fig. 2A,D). These results reflected the successful transfection of miR‐93‐3p mimic and inhibitor.

**Figure 2:** Transfection efficiency of pcDNA‐ZNF667‐AS1, si‐ZNF667‐AS1, and miR‐93‐3p mimic and inhibitor in HeLa and C‐33A cells was measured by RT/qPCR. (A–C) The transfection efficiency of pcDNA‐ZNF667‐AS1 and si‐ZNF667‐AS1 in HeLa cells. (D–F) The transfection efficiency of pcDNA‐ZNF667‐AS1 and si‐ZNF667‐AS1 in the C‐33A cells. (A, D) The expression of miR‐93‐3p was remarkably increased in the cells transfected with miR‐93‐3p mimic, but obviously decreased in the cells transfected with miR‐93‐3p inhibitor. (B, E) The cells transfected with pcDNA‐ZNF667‐AS1 showed increased expression of ZNF667‐AS1 in a concentration‐dependent manner. (C, F) The cells transfected with si‐ZNF667‐AS1 showed decreased expression of ZNF667‐AS1 in a concentration‐dependent manner. The data were expressed as mean ± standard deviation. The experiment was independently repeated three times. Comparisons among multiple groups were performed by ANOVA, followed by Tukey *post hoc* test. *P < 0.05 vs. the vector group. ^#^ *P* < 0.01 vs. the si‐NC group.

Upon transfection of HeLa and C‐33A cells with pcDNA‐ZNF667‐AS1 and si‐ZNF667‐AS1 each, the cells transfected with pcDNA‐ZNF667‐AS1 showed an increased expression of ZNF667‐AS1 in a concentration‐dependent manner (*P* < 0.05, Fig. 2B,E). We designed and transfected three ZNF667‐AS1 silencing sequences (Table S1) and found that the interference efficiency of si‐ZNF667‐AS1 with siRNA‐1 and siRNA‐3 sequences was significant (*P* < 0.05), among which the interference efficiency of siRNA‐1 was highly significant (*P* < 0.005), while that of siRNA‐2 was not significant (*P *> 0.05; Fig. 2C,F). These findings were indicative of successful plasmid‐induced intervention in ZNF667‐AS1 expression. Therefore, 2 μg·mL^−1^ pcDNA‐ZNF667‐AS1 and 20 μm si‐ZNF667‐AS1 were selected for the subsequent experiments.

### 3.3 Upregulation of ZNF667‐AS1 attenuates cell cycle entry and invasion of CC cells

Transwell assay and flow cytometry were employed to assess the effects of ZNF667‐AS1 on cell invasion and cell cycle distribution of HeLa (Fig. 3A–D) and C‐33A (Fig. 3E–H) cells. In comparison with the control and vector groups, ZNF667‐AS1 elevation decreased cell invasion and the proportion of cells in the S phase, while elevating the proportion of cells in the G1 phase (*P* < 0.05). In comparison with the control and ctrl siRNA groups, si‐ZNF667‐AS1 increased cell invasion and the proportion of cells in the S phase as well as in the G1 phase (*P* < 0.05). Collectively, the results demonstrated that upregulation of ZNF667‐AS1 suppressed cell invasiveness and cell cycle entry in HeLa and C‐33A cells.

**Figure 3:** Transwell assay and flow cytometry showed that the repression of ZNF667‐AS1 expression induced invasion and cell cycle entry of HeLa and C‐33A cells. (A–D) The results of HeLa cells. (E–H) The results of C‐33A cells. (A, E) Transwell assay was used to assess the effects of ZNF667‐AS1 on cell invasion (×200, scale bar = 50 μm). (B, F) Repression of ZNF667‐AS1 expression could enhance the invasion of HeLa and C‐33A cells. (C, G) PI staining was performed to evaluate cell cycle distribution in HeLa and C‐33A cells. (D, H) Repression of ZNF667‐AS1 expression could promote cell cycle entry in HeLa and C‐33A cells. The data were expressed as mean ± standard deviation. The experiment was independently repeated three times. Comparisons among multiple groups were performed by ANOVA, followed by Tukey *post hoc* test. *P < 0.05 vs. the control group.

### 3.4 ZNF667‐AS1 competitively binds to miR‐93‐3p to upregulate PEG3 in CC cells

Fluorescence *in situ* hybridization was employed to determine the subcellular localization of ZNF667‐AS1 in HeLa cells. As shown in Fig. 4A, the cell nuclei were stained blue by DAPI while ZNF667‐AS1 was stained red. In the ZNF667‐AS1 group, ZNF667‐AS1, stained in red, was primarily localized in the cytoplasm as compared to the control group. These findings signified that ZNF667‐AS1 was principally localized in the cytoplasm of HeLa cells, which suggested that ZNF667‐AS1 might function as a ceRNA. As shown in Fig. 4B, compared with the cells without transfection, luciferase activity was significantly decreased upon cotransfection with miR‐93‐3p mimic and ZNF667‐AS1‐Wt (*P* < 0.05). No significant difference in luciferase activity was observed after cotransfection with miR‐93‐3p and ZNF667‐AS1‐Mut (*P *> 0.05). These findings are indicative of a target‐gene relationship of ZNF667‐AS1 with miR‐93‐3p. As shown in Fig. 4C, miR‐93‐3p had a target relationship with PEG3. Competitive binding between ZNF667‐AS1 and miR‐93‐3p was confirmed with the RNA pull‐down experiment. In comparison with the Bio‐probe‐NC group, ZNF667‐AS1 was markedly enriched in the Bio‐miR‐93‐3p‐Wt group (*P* < 0.05), while no significant difference was observed in the Bio‐miR‐93‐3p‐Mut group (*P *> 0.05; Fig. 4D). These results demonstrated that ZNF667‐AS1 could specifically bind to miR‐93‐3p. As shown in Fig. 4E, miR‐93‐3p could specifically bind to PEG3. After overexpressing or silencing ZNF667‐AS1, ZNF667‐AS1 was found to downregulate miR‐93‐3p and upregulate PEG3 (Fig. 4F). After overexpressing or silencing miR‐93‐3p, it was evident that miR‐93‐3p downregulated ZNF667‐AS1 and PEG3 (Fig. 4G). Figure 4A–G showed the results of the experiments performed in HeLa cells. In addition, we repeated experiments in C‐33A cells (Fig. 4H–N), and the results in these two cell lines were consistent. These findings conclusively demonstrated that the competitive binding of ZNF667‐AS1 to miR‐93‐3p could regulate the expression of PEG3 in CC cells.

**Figure 4:** Mutual regulation and competitive binding of miR‐93‐3p to ZNF667‐AS1 were verified, which regulates PEG3 in CC. (A–G) The experiment results of HeLa cells, (H–N) show the experiment results of C‐33A cells. (A, H) ZNF667‐AS1 location in HeLa and C‐33A cells detected by FISH assay (×400, scale bar = 25 μm). (B, I) miR‐93‐3p binds to ZNF667‐AS1 in its 3′UTR. ZNF667‐AS1‐Wt and ZNF667‐AS1‐Mut were cotransfected with miR‐93‐3p mimic into HeLa and C‐33A cells, followed by dual‐luciferase reporter assay to identify the regulatory relationship between ZNF667‐AS1 and miR‐93‐3p. *P < 0.05 vs. the NC group. (C, J) miR‐93‐3p binds to PEG3 in its 3'UTR. PEG3‐Wt and PEG3‐Mut were cotransfected with miR‐93‐3p mimic into HeLa and C‐33A cells, followed by dual‐luciferase reporter assay to identify the regulatory relationship between PEG3 and miR‐93‐3p. *P < 0.05 vs. the NC group. (D, K) RNA pull‐down assay showed that the expression of ZNF667‐AS1 was markedly increased in the Bio‐miR‐93‐3p‐Wt group than that in the Bio‐probe‐NC group. *P < 0.05 vs. the Bio‐probe‐NC group. (E, L) RNA pull‐down assay showed that the expression of PEG3 was markedly increased in the Bio‐miR‐93‐3p‐Wt group than that in the Bio‐probe‐NC group. *P < 0.05 vs. the Bio‐probe‐NC group. (F, M) relative expression of miR‐93‐3p and PEG3 was measured using RT/qPCR, which indicated that miR‐93‐3p expression was increased and PEG3 expression was decreased when cells treated with si‐ZNF667‐AS1. *P < 0.05 vs. the oe‐NC group. ^#^ *P* < 0.05 vs. the si‐NC group. (G, N) Relative expression of ZNF667‐AS1 and PEG3 was determined by RT/qPCR, which indicated that ZNF667‐AS1 and PEG3 expression was increased when cells treated with miR‐93‐3p inhibitor. In G, *P < 0.05 vs. the NC group. In N, *P < 0.05 vs. the NC‐mimic group; ^#^ *P* < 0.05 vs. the NC inhibitor group. The data were expressed as mean ± standard deviation. The experiment was independently repeated three times. Data between two groups were compared by independent sample *t*‐test, and comparisons among multiple groups were performed by ANOVA, followed by Tukey *post hoc* test.

### 3.5 ZNF667‐AS1 negatively regulates miR‐93‐3p and inhibits cell invasion and cycle *via* PEG3

The aforementioned findings revealed the regulatory mechanism involving ZNF667‐AS1, miR‐93‐3p, and PEG3, leading to the investigation of the effects of their interaction on the cell cycle and invasion in HeLa cells (Fig. 5A–J) and C‐33A cells (Fig. 5K–T). Transfection with pcDNA‐ZNF667‐AS1 increased the expression of ZNF667‐AS1, PEG3, and TIMP‐2, while reducing the cell invasion capability and expressions of miR‐93‐3p, MMP‐2, and MMP‐9, in contrast to cells without transfection (all *P* < 0.05; Fig. 5A–E and Fig. 5K–O). However, si‐ZNF667‐AS1 transfection reduced the expression of ZNF667‐AS1, PEG3, and TIMP‐2, increased the expression of miR‐93‐3p, MMP‐2, and MMP‐9, and also promoted cell invasion (all *P* < 0.05). No significant differences in the expression of ZNF667‐AS1, miR‐93‐3p, PEG3, TIMP‐2, MMP‐2, and MMP‐9 and cell invasion capability were observed after the cells were cotransfected with si‐ZNF667‐AS1 and miR‐93‐3p inhibitor (all *P *> 0.05). The expression of PEG3 and TIMP‐2 increased in cells cotransfected with si‐ZNF667‐AS1 and miR‐93‐3p inhibitor, while the cell invasion capability and the expression of miR‐93‐3p, MMP‐2, and MMP‐9 decreased in these cells (all *P* < 0.05). These results signified that ZNF667‐AS1 negatively regulated miR‐93‐3p, which in turn reversed PEG3 attenuation and HeLa cell invasion triggered by reduced ZNF667‐AS1.

**Figure 5:** ZNF667‐AS1 inhibited miR‐93‐3p expression and suppressed cell cycle and invasion of HeLa and C‐33A cells. (A–J) show the results of HeLa cells while (K–T) show the results of C‐33A cells. (A, K) RT/qPCR demonstrated that ZNF667‐AS1 elevation decreased the expression of miR‐93‐3p, MMP‐2 mRNA, and MMP‐9 mRNA, and increased the expression of PEG3 and TIMP‐2 mRNAs. (B, L) The protein bands of MMP‐2, MMP‐9, PEG3, and TIMP‐2 in western blot analysis after the cells were transfected with pcDNA‐ZNF667‐AS1 and si‐ZNF667‐AS1. (C, M) Western blot analysis demonstrated that ZNF667‐AS1 elevation decreased the protein levels of MMP‐2 and MMP‐9, and increased the protein levels of PEG3 and TIMP‐2. (D, N) Images of migrated cells in Transwell assay after the cells were transfected with pcDNA‐ZNF667‐AS1 and si‐ZNF667‐AS1 (×200, scale bar = 50 μm). (E, O) Transwell assay results showed that ZNF667‐AS1 elevation inhibited cell invasion, while ZNF667‐AS1 silencing enhanced cell invasion. (F, P) RT/qPCR demonstrated that ZNF667‐AS1 elevation decreased the expression of miR‐93‐3p and cyclin D1 mRNA, and increased the expression of PEG3 and p16 mRNAs. (G, Q) The protein bands of cyclin D1, PEG3, and p16 in western blot analysis after the cells were transfected with pcDNA‐ZNF667‐AS1 and si‐ZNF667‐AS1. H and R, western blot analysis demonstrated that ZNF667‐AS1 elevation decreased the protein level of cyclin D1 and increased the protein levels of PEG3 and p16. I and S, Flow cytometry results of cell cycle distribution after the cells were transfected with pcDNA‐ZNF667‐AS1 and si‐ZNF667‐AS1. (J, T) Flow cytometry showed that ZNF667‐AS1 elevation inhibited cell cycle entry, while ZNF667‐AS1 silencing promoted cell cycle entry. Data are presented as mean ± standard deviation. The experiment was independently repeated three times. Comparisons among multiple groups were performed by ANOVA, followed by Tukey *post hoc* test. *P < 0.05 vs. the control group.

pcDNA‐ZNF667‐AS1 transfection increased the expression of ZNF667‐AS1, PEG3, and p16 and the proportion of cells in the G1 phase, while reducing the proportion of cells in the S phase and the expression of miR‐93‐3p and cyclin D1 when compared to the cells without transfection (all *P* < 0.05). On the contrary, si‐ZNF667‐AS1 reduced the expression of ZNF667‐AS1, PEG3, and p16 and the proportion of cells in the G1 phase, while it increased the proportion of cells in the S phase and the expressions of miR‐93‐3p and cyclin D1 (all *P* < 0.05). No significant differences in the expression of ZNF667‐AS1, miR‐93‐3p, PEG3, cyclin D1, and p16 and cell cycle distribution were observed after cotransfection with si‐ZNF667‐AS1 and the miR‐93‐3p inhibitor (all *P *> 0.05). In addition, the expression of ZNF667‐AS1, PEG3, and p16 and the proportion of cells in the G1 phase increased in the cells cotransfected with si‐ZNF667‐AS1 and miR‐93‐3p inhibitor, while the proportion of cells in the S phase and the expression of miR‐93‐3p and cyclin D1 in these cells had decreased (all *P* < 0.05). These findings similarly demonstrated that ZNF667‐AS1 negatively regulated miR‐93‐3p, and the downregulation of miR‐93‐3p could in turn reverse the repression of PEG3 and cell cycle entry triggered by the reduced expression of ZNF667‐AS1 (Fig. 5F–J,P–T).

### 3.6 Upregulated ZNF667‐AS1 or downregulated miR‐93‐3p inhibits tumor growth and metastasis in nude mice

To verify the results of *in vitro* experiments, the effects of ZNF667‐AS1 and miR‐93‐3p on tumor formation in nude mice were evaluated using a tumor xenograft model (Fig. 6 and Table 2). As Fig. 6A–C shows, in comparison with the control group, the volume and weight of tumors were decreased in the ZNF667‐AS1 vector group, but increased in the si‐ZNF667‐AS1 group (all *P* < 0.05). No significant differences in the volume and weight of tumors were observed between the control and the si‐ZNF667‐AS1 + miR‐93‐3p inhibitor groups (*P *> 0.05). Moreover, as shown in Table 2 and Fig. 6D–E, the number of metastatic lymph nodes was markedly decreased in the ZNF667‐AS1 vector group in conjunction with an increased expression of MTA‐1, whereas number of metastatic lymph nodes was increased in the si‐ZNF667‐AS1 group in conjunction with a lower expression of MTA‐1 (all *P* < 0.05). The results of *in situ* hybridization revealed that ZNF667‐AS1 expression was increased and miR‐93‐3p expression was deceased in xenograft tumors tissue of mice in the ZNF667‐AS1 vector group, as compared to the control group, which was opposite in the si‐ZNF667‐AS1 group (all *P* < 0.05). The expression of ZNF667‐AS1 and miR‐93‐3p did not differ greatly in the si‐ZNF667‐AS1 + miR‐93‐3p inhibitor group (*P *> 0.05; Fig. 6F–G). These findings demonstrated that downregulation of miR‐93‐3p could reverse the simulative effect of reduced ZNF667‐AS1 expression on tumor metastasis. Overall, it was evident that ZNF667‐AS1 negatively regulated miR‐93‐3p, and the downregulation of miR‐93‐3p reversed tumorigenesis and metastasis promotion triggered by a reduced expression of ZNF667‐AS1.

**Figure 6:** *In vivo* experiments indicated that downregulated ZNF667‐AS1 expression or upregulated miR‐93‐3p expression promoted tumor growth and metastasis in nude mice. (A) The tumor growth curve in nude mice after transfection of pcDNA‐ZNF667‐AS1, si‐ZNF667‐AS1 and miR‐93‐3p inhibitor. (B) Nude mice and their tumor tissues on the 15th day after transfection with pcDNA‐ZNF667‐AS1, si‐ZNF667‐AS1, and miR‐93‐3p inhibitor. (C) Compared with the control group, the tumor weight on the 15th day was decreased in the ZNF667‐AS1 vector group, but increased in the si‐ZNF667‐AS1 group. (D) Positive MTA‐1 expression in nude mice after inoculation with pcDNA‐ZNF667‐AS1, si‐ZNF667‐AS1, and miR‐93‐3p (×400, scale bar = 25 μm). (E) Immunohistochemistry analysis of positive expression of MTA‐1 protein. (F) Images of *in situ* hybridization of the tumor tissues (×400, scale bar = 25 μm). (G) Quantitative analysis of the *in situ* hybridization results. Data are presented as mean ± standard deviation. Comparisons among multiple groups were performed by ANOVA, followed by Tukey *post hoc* test. Comparison of tumor volume in different mice was analyzed by repeated measurement ANOVA. *n* = 8. ^*^ *P* < 0.05 vs. the control group.

**Table 2:** The lymph node metastasis in nude mice after inoculation of pcDNA‐ZNF667‐AS1, si‐ZNF667‐AS1, or miR‐93‐3p. si‐ or siRNA, small interfering RNA. *n* = 8. Metastatic lymph nodes were compared by ANOVA. *P < 0.05, vs. the control group.

Group	Mice	Metastatic lymph nodes	Metastasis rate (%)
Control	8	8.57 ± 0.79	72
ZNF667‐AS1 vector	8	3.12 ± 0.27*	24
si‐ZNF667‐AS1	8	11.86 ± 0.93*	90
si‐ZNF667‐AS1 + miR‐93‐3p inhibitor	8	7.96 ± 0.74	69

## 4 Discussion

Cervical cancer has remained a persistent cause of high mortality in women worldwide, with diagnosis commonly achieved at later invasive stages, leading to poor treatment and prognosis (Cancer Genome Atlas Research *et al.*, 2017). The invasion and metastasis of cancer cells could be problematic for the diagnosis and poor prognosis (He *et al.*, 2012). Identifying their molecular processes is an unmet need, with the potential to facilitate improved treatment for CC patients. Recently, ZNF667‐AS1, an lncRNA, was found to have an anticarcinogenic role in CC (Zhao *et al.*, 2017). The current study aimed to study and elucidate the role of the ZNF667‐AS1/miR‐93‐3p/PEG3 axis in CC.

Initially, the data obtained from the current study demonstrated that ZNF667‐AS1 and PEG3 were poorly expressed, while miR‐93‐3p was found to be abundant in CC tissues. Online software analysis and cell‐based experiments signified the mutual regulation and competitive combination between ZNF667‐AS1 and miR‐93‐3p. ZNFs are a superfamily of transcription factors, which are abundantly expressed in eukaryotic cells (Nie *et al.*, 2016). Multiple ZNFs have been investigated with regard to CC. Overexpression of the ZNF; ZNF268b2 has been linked to NF‐κB activation leading to CC carcinogenesis (Wang *et al.*, 2012). Huang *et al.* have identified the possible efficacy of hypermethylated ZNF582 in the molecular measurement of CC. Our results are consistent with a previous report of ZNF667‐AS1 downregulation in CC tissues (Zhao *et al.*, 2017). Further investigation into the functional and regulatory roles played by ZNFs in CC is essential to provide biological insight. The pattern of competitive combination between ZNFs and miRNAs has been noted in many reports. Anticancer ZNF238 is repressed by miR‐20b overexpression whereas ZNF24, a tumor promoter, is increased by miR‐940 dysregulation (Lu *et al.*, 2015). In clear cell renal cell carcinoma cells, miR‐93‐3p was found to decrease the expression of pigment epithelium‐derived factor (PEDF) and inhibit osteogenesis (Wang *et al.*, 2017). As a single miRNA can distinctively alter the expression of multiple mRNA transcripts (Hu *et al.*, 2010; Li *et al.*, 2010), we hypothesized that miR‐93‐3p dysregulation is closely related to CC cell behavior. We verified PEG3 as a target of miR‐93‐3p, which is localized on the human chromosome 19q13.4/proximal mouse chromosome 7 (Perera and Kim, 2016) and is close to the locations of many zinc finger genes (Lleras *et al.*, 2011). The C2H2 zinc finger domain functions in DNA binding, whereas the KRAB‐A domain is responsible for the physical interaction and subsequent recruitment of KRAB‐ZFP‐associated protein 1 (KAP1) (Brayer and Segal, 2008; Groner *et al.*, 2010). A previous report found ZBRK1 silencing occurring *via* KAP1 enhanced CC metastasis and invasion (Lin *et al.*, 2013). PEG3 was previously reported to inhibit downstream transcription of ZNF proteins through its interaction with the corepressor KAP1 (He and Kim, 2014). Furthermore, DNA methylation at PEG3 has been considered as a susceptibility locus for transition of cervical intraepithelial neoplasia to invasive CC (Nye *et al.*, 2013). These reports appear consistent with our finding that PEG3 acted as a tumor suppressor in CC.

The present study also demonstrated that, *via* PEG3, upregulated miR‐93‐3p expression and downregulated ZNF667‐AS1 expression could promote the invasion of CC cells and its cell cycle entry. The p53 apoptosis pathway may inhibit growth or induce cell death, while PEG3 functions downstream of p53 by stimulating apoptosis through interactions with Bax (Broad *et al.*, 2009; Nye *et al.*, 2013). MMP‐2 and MMP‐9 are known to critically function in tumor invasion and metastasis and have been speculated as effective targets for CC treatment (Roomi *et al.*, 2010). In the Burkitt's lymphoma cell line, both MMP‐2 and MMP‐9 exercised their functions under the modulation of PEG10 (Xiong *et al.*, 2012). Von and colleagues reported p16 as a robust biomarker for the prevention of CC or other HPV‐related cancers (von Knebel Doeberitz *et al.*, 2012). Cyclin D1 activation has been associated with epidermal growth factor‐stimulated human CC cell growth (Narayanan *et al.*, 2012). A high level of MTA1 protein is linked to enhanced lymph node metastasis and increased risk of CC recurrence, thus potentiating its clinical significance in future gene‐targeted therapies for CC patients (Liu *et al.*, 2013). At the cellular level, MTA1 also promotes CC cell growth, invasion, migration, as well as adhesion and colony formation (Han *et al.*, 2011). In addition, downregulation of MTA2 is involved in proper imprinted expression of PEG3 gene (Ma *et al.*, 2010). Taken together, these prior reports support our conclusion that upregulation of ZNF667‐AS1 and consequent repression of miR‐93‐3p enhance the expression of PEG3, which consequently increases the concentrations of p16 and TIMP‐2 while reducing MMP‐2/‐9 concentration. Ultimately, these changes decrease the cell cycle entry, invasion, and metastasis of CC. Our *in vivo* experiments also indicated that overexpressed ZNF667‐AS1 inhibited tumor growth and metastasis.

## 5 Conclusion

In conclusion, lncRNA ZNF667‐AS1 decreased the cell cycle entry, invasion, and metastasis of CC by inhibiting the expression of miR‐93‐3p and upregulating the expression of PEG3 (Fig. 7). Therefore, the identification of ZNF667‐AS1/miR‐93‐3p/PEG3 axis in the invasion and metastasis of CC may provide an insight in understanding the mechanisms of CC. Future studies with larger cohort experiments are needed to clarify the detailed mechanisms of ZNF667‐AS1/miR‐93‐3p/PEG3 in CC. Meanwhile, future mechanistic studies should be more scrupulously and logically performed in diverse populations, in order to further the promising direction revealed by the current findings.

**Figure 7:** Schematic diagram of the regulation of ZNF667‐AS1 in CC. ZNF667‐AS1 negatively regulated miR‐93‐3p expression by targeting PEG3, thereby restraining cell proliferation and EMT. PEG3 increased the expression of TIMP‐2 and p16, and further decreased the expression of MMP‐2 and MMP‐9.

## Conflict of interest

The authors declare no conflict of interest.

## Author contributions

YJL and YW designed the study. ZY, YYW, and YW collated the data, carried out data analyses, and produced the initial draft of the manuscript. YJL, ZY, and YYW contributed to drafting the manuscript. All authors have read and approved the final submitted manuscript.

## Supporting information


**Table S1**. Sequences of three siRNAs of ZNF667‐AS1.
